This article has been retracted.

# Histopathological Investigations and Molecular Confirmation Reveal *Mycobacterium bovis* in One-Horned Rhinoceros (*Rhinoceros unicorns*)

**DOI:** 10.1155/2022/5816986

**Published:** 2022-05-18

**Authors:** Abu Baker Siddique, Riaz Hussain, Adil Jamal, Md. Belal Hossain, Zulfiqar Ahmad, Muhammad Khalid Mansoor, Iahtasham Khan, Kainat Zahra, Ahrar Khan

**Affiliations:** ^1^Department of Microbiology, Government College University, Faisalabad, Pakistan; ^2^Department of Pathology, Faculty of Veterinary and Animal Sciences, The Islamia University of Bahawalpur, 63100, Pakistan; ^3^Sciences and Research, College of Nursing, Umm Al Qura University, 715 Makkah, Saudi Arabia; ^4^Department of Plant Pathology, Faculty of Agriculture, Sher-e-Bangla Agricultural University, Sher-e-Bangla Nagar, Dhaka 1207, Bangladesh; ^5^Department of Food Science and Technology, Faculty of Agriculture and Environment, Baghdad-Ul-Jadeed Campus, The Islamia University of Bahawalpur-63100, Pakistan; ^6^Department of Microbiology, Faculty of Veterinary and Animal Sciences, The Islamia University of Bahawalpur, 63100, Pakistan; ^7^Section of Epidemiology and Public Health, University of Veterinary and Animal Sciences, Lahore, Sub-Campus Jhang, Pakistan; ^8^Institute of Biochemistry and Biotechnology, University of Veterinary and Animal Sciences, Lahore, Pakistan; ^9^Shandong Vocational Animal Sciences and Veterinary College, Weifang 261061, China; ^10^Faculty of Veterinary Science, University of Agriculture, Faisalabad, Pakistan

## Abstract

*Mycobacterium bovis* causes tuberculosis in dairy and wild animals. Presence of tuberculosis in animals poses a threat not only to their herd mates but also for public. No reports are available about the clinical, pathological, and molecular investigation of naturally occurring tuberculosis (TB) due to *M. bovis* in one-horned rhinoceros. One-horned female rhinoceros (*Rhinoceros unicorns*) at the age of 41 years died in a public park in Pakistan. Postmortem and other investigations were carried out to know the cause of death. The present study describes necropsy, histopathology, and molecular-based confirmation of TB in a captive female rhinoceros that died of this infection. Clinically, the rhinoceros showed nonspecific clinical signs including anorexia, lethargy, dyspnoea, coughing, and sudden death. At necropsy, the trachea exhibited mild congestion and contained catarrhal exudate at the bronchial bifurcation. Macroscopic examination revealed characteristic tubercles on all parenchymatous organs. The lungs showed consolidation, grey hepatization, and contained granulomatous lesions packed with cheesy exudate. Histopathological examination showed severe pneumonic changes in the form of granulomatous inflammation consisting of lymphocytes, multinucleated giant cells, caseous materials, and mineralized foci surrounded by a fibrous capsule. PCR amplicon of 500 bp confirmed the presence of *M. bovis* in multiple hepatic and pulmonary tissue samples, as well as in uterine exudates. It was concluded that the presence of tuberculosis in rhinoceros may pose potential transmission risk to other animals and the application of practical tools to determine TB status in the rhinoceros is crucial.

## 1. Introduction

Tuberculosis (TB) produced by *Mycobacterium tuberculosis* is an infectious and chronic debilitating illness that affects humans, domestic animals, and wild animals worldwide [1]. *M. tuberculosis* is the most important pathogen causing human tuberculosis, whereas *Mycobacterium bovis* is the most important pathogen causing bovine tuberculosis (BTB) and has a high potential to infect humans and other animals due to its wide host range [2]. Because of its occurrence in numerous animal species and their products, which are utilized for human consumption, this disease is of significant economic and public health importance [3]. Several developed countries have recently reduced or eliminated BTB from their cattle populations, but significant pockets of infection remain in developing countries of world in wildlife [4]. Several investigations regarding have been reported in large and small ruminants in Pakistan [5].

Transmission of *M. bovis* to public health mainly occurs through inhalation, consumption of untreated milk/raw milk, aerosols inhalation of the pathogen from morbid animals at the time of close contact, and shedding of bacteria by infected animal for the environmental contamination [6]. The exact transmission of the infectious agent to wildlife animals is still not clear. The acquisition of infected animals, herd size, poor husbandry, and sanitary procedures is the key routes of disease transfer into herds. Furthermore, animal herds with a stronger tendency to roam play an important role in disease transmission [6]. However, different studies have reported that the infected dairy animals and wild animals secrete *M. bovis* in their faeces and urine, as bacilli have been detected in naturally contaminated environmental samples such as soil and faeces [7].

*M. bovis* has proven to infect multiple hosts within the wildlife community [8]. Data on human tuberculosis due to *M. bovis* is poorly documented [9]. Different studies have reported various risk factors with tuberculosis in cattle and buffaloes kept at various livestock farms [9]. Specific data on bovine tuberculosis in Pakistan's wild animals are scarce except few reports in zoo animals [10]. *M. tuberculosis* and *M. bovis* have been found in black rhinoceros confined in zoos or under semi-intensive management [11]. Despite the presence of *M. bovis* in livestock and other wildlife species in Pakistan with rhinoceros populations, no instances of tuberculosis have been observed in rhinos.

TB is often diagnosed by isolating the organism from sputum, milk, faeces, and other body fluids [12]. The usual methods for diagnosing tuberculosis include direct smear microscopy using the fluorescent acid-fast staining technique and Ziehl-(ZN) Neelsen's staining of clinical samples [12]. Although cultivation on selective media offers a confirmed diagnosis of Mycobacterium but the primary disadvantage of this method is the slow bacterial growth [13]. Rapid diagnosis of Mycobacterium from clinical samples is possible using polymerase chain reaction (PCR) amplification of the Mycobacterial DNA. PCR is a more precise and reliable approach for quick diagnosis with much more sensitivity and specificity comparable to bacterial culture [13].

Our study aimed to study necropsy lesions followed by histopathological findings of tuberculosis due to *M. bovis* in a captive female rhinoceros. *M. bovis* detection was further confirmed based on molecular approach using PCR. Regular livestock and wildlife screening will help to prevent *M. bovis* transmission to other animals.

## 2. Materials and Methods

### 2.1. Ethical Statement

The technical and ethical committee constituted by Department of Pathology, Faculty of Veterinary and Animal Sciences, The Islamia University of Bahawalpur, Pakistan, approved the protocol of the postmortem study of one-horned rhinoceros.

### 2.2. Study Area and Sample

South Punjab region had tropical and subtropical climatic conditions with hot and humid summer and cold winter. In this region, lack of intensive animal health monitoring facilities, nutrition, water sources, and unavailability of sufficient seasonal fodder are the main limitations for the livestock and various other animals. Near the zoological park where the rhinoceros was kept, the region is mainly dominated by nomadic and sedentary system where the animals are routinely migrated for fodder and water which may cause spread of infectious agents from one location to other during common grazing and drinking.

At that time, these animals were transported on the recommendations of the governor of Punjab to district Bahawalpur and were kept at Lal Suhanra National Park Punjab province. The administrator of the park built a trench-cum-lake where these animals were kept. The rhinoceros were daily monitored for any obvious clinical ailments. According to the administration of the Park and history from the caretakers, female rhinoceros was feed green seasonal fodder (90 kg), bread (5 kg), and mixed grains (4 kg), daily. According to the administrator of park, the female might have died because of excessive bleeding that had weakened her. The veterinary assistants of the park noted animal stillbirth in rhinoceros. Animal became sick, showing nonspecific signs such as depression, anorexia, lethargy, disorientation, dyspnoea, and coughing. Despite treatment, the rhinoceros died asymptomatically in December 2019.

### 2.3. Necropsy Examination

The necropsy was performed soon after death. Before complete skinning, the animal was carefully examined for external lesions. The rhinoceros was average and fair in body condition. However, congested nasal mucosa, pale mucous membrane, and bloody discharge from the vagina were observed. Afterward, a complete postmortem examination was performed [14].

### 2.4. Sample Collection and Histopathological Analysis

Morbid tissues exhibiting lesions, including lungs and liver, were collected and fixed in 10% neutral buffered formalin for microscopic investigation. Tissues were embedded in paraffin wax, and sections of about 4-5 *μ*m thick were cut [15] and stained with hematoxylin and eosin stain for histopathological examination.

### 2.5. Genomic DNA Extraction and Molecular Detection

For bacilli detection and confirmation, various tissue samples having lesions, e.g., liver, lungs, and uterine pus were used for bacterial DNA extraction and confirmation of suspected cause. Genomic DNA was extracted from samples using GeneJET Genomic DNA Extraction kit (Thermo Scientific, USA). The species-specific primer targeting the JB21 and JB22 genes (forward JB21; 5′-TCGTCCGCTGATGCAAGTGC-3′, reverse JB22; 5′-CGTCCGCTGACCTCAAGAAG-3′) were used for the confirmation of samples [16]. The amplification conditions were set as initial denaturation at 95°C for 4 min followed by 30 cycles of denaturation at 94°C for 1 min, annealing at 55°C for 30 s, and primer extension at 72°C for 1 min, with a final extension at 72°C for 10 min. The amplification was performed using PCR master mixture (2X) (Cat # 0171, Invitrogen, USA) and thermocycler (T 100 Thermal cycler, BioRad, USA). The PCR product was run on 1% agarose gel for electrophoreses and visualized through gel documentation system (Gel Doc XR+ System, BioRad, USA).

## 3. Results

In the present study, at necropsy, the external examination showed that the female rhinoceros was normal and had fair body condition. The carcass exhibited congested nasal mucosa, pale mucous membrane, and bloody discharge from the vagina (Figure 1(a)). The head, skin, eyes, mouth, ears, and rectum appeared normal. After skinning, the abdominal cavity exhibited moderate hyperaemia of serosal membranes and mild peritonitis. The small and large intestines showed moderated ballooning and appeared empty. The external surfaces of the rectum appeared hyperaemic. The spleen was moderately hyperaemic. The reproductive organs showed severe inflammatory changes, including metritis and pyometra. The inner surfaces of the uterus were thick and contained pus mixed with tissue debris (Figure 1(b)).

The trachea showed mild congestion and contained catarrhal exudates at the bifurcation junction. The thoracic cavity showed moderate pleural adhesions. The lungs exhibited grey hepatization, consolidation, and granulomatous lesions. Lesions in the lungs were small multifocal tubercular lesions containing creamy white caseous material exudate (Figure 1(c)). The liver was found consolidated, hyperaemic, dark in color, enlarged, and had tuberculous nodules packed with caseous material (Figure 1(d)).

Histopathological examination of lungs exhibited fibrino-necrotic edema, thickening of interlobular septa with infiltration of chronic inflammatory cells, and ruptured interalveolar septa (Figure 2(a)). Fibrosis, hyperplasia of pneumocytes, the punctuation of mononuclear cells, and multinucleated giant cells in alveolar spaces obliterating the adjacent alveoli were also seen (Figure 2(b)). Extensive micro and macrotubercular nodules with exudate surrounded by fibroblast fronts, fibrocytes, monocytes, macrophages, and caseous and calcified material were seen in the lamellar arrangement (Figures 2(b)–2(d)). Multiple granulomatous foci contain fibrosis, bacilli, and lymphohistiocytic inflammatory cells (Figure 3(a)). Histopathological observation of liver sections showed immature and mature tubercles, heavily infiltrated with inflammatory cells in portal triad areas. Perivascular cuffing of lymphocytes, monocyte, and fibroblasts was seen. Numerous small blood-filled angiomatous cysts were observed. Bilateral granulomatous inflammation and bronchial exudate were the consistent findings in infected lungs. The PCR (500pb) confirmed *M. bovis* in samples collected from the liver, lungs, and uterine pus (Figure 3(b)). We did not observe lesions in mesenteric lymph nodes in this case. Therefore, mesenteric lymph nodes were not obtained.

## 4. Discussion

Tuberculosis is a highly contagious zoonotic disease transmitted to wild animals in captivity in close contact with free-ranging animals [17]. Wild animals are susceptible to tuberculosis and can act as reservoirs, maintain the infectious agents, and continued the spill over of the disease via scavenged carcasses or by prey. In the present study, we reported the *M. bovis* based mortality in rhinoceros in southern Punjab region, Bahawalpur, Pakistan. The researchers discovered tuberculous lesions in rhinoceros, which was consistent with prior investigations in other animals [18, 19, 20, 21] but rarely reported than other findings [23, 24]. The prevalence of TB varies from country to country, or even within a country [22]. This variation might be linked to the type of animal production system [23, 24] and animal breed [25]. Tuberculous lesions have also been seen in parenchymatous organs of slaughtered animals [12] and in an adult female Marsican brown bear died due to *M. bovis* infection [26].

The diagnosis of TB in wild animals mainly relies on necropsy lesions, histopathology, and the bacterial culturing. The changes and distribution of lesions caused by *M. bovis* mainly depend upon the possible route of infection. Very few information is available about the gross and microscopic lesions due to *M. bovis* in captive individuals' rhinoceroses [27, 28] and very rare in free-ranging wild animals. Similar pulmonary lesions have been seen in a semicaptive black rhinoceros due to natural infection with *M. bovis* [29]. However, no characteristic lesions have been observed in rhinoceros experimentally infected with *M. bovis* [27].

Bilateral granulomatous inflammation and bronchial exudate were the consistent findings in infected lungs in the present case. It is speculated that in *M. bovis*, infected lungs caseated tissues liquefy due to the liberation of nucleases and proteases from macrophages [7]. Lungs of dairy cattle infected with *M. bovis* showed frequent classical lesions of tuberculosis, such as granuloma comprising caseation/mineralization surrounded by epithelioid, multinucleated giant cells, fibrous capsule, plasma cells, and lymphocytes [7, 12]. Similarly, granulomatous inflammation composed of mixed inflammatory cells, multinucleated giant cells, fibrous nodules, and mineralized centers has been observed in the lungs of experimentally induced *M. bovis* infection in rhinoceros [27]. No report is available in the accessible published literature about the presence of blood-filled cysts in the liver of rhinoceroses due to *M. bovis* infection. However, it has been observed in the liver of crossbred cows suffered from chronic tuberculosis [7].

PCR assays are the most promising alternative tool for the quick and specific detection of tuberculosis [30, 31, 32]. PCR techniques have been effectively utilized to diagnose bovine tuberculosis in a variety of naturally infected organic samples, including tissue, blood, and nasal exudates [32, 33]. The most widely used method is based on primers that amplify parts of the DNA. JB21/JB22 has been shown to be extremely accurate at identifying *M. bovis* DNA isolates from blood samples, with 100 percent concordance with the traditional microbiological approach [34]. Studies reported in past also employed a multiplex-PCR to detect a single 500 bp product in *M. bovis* while MTB produced a single 185 bp product, with or without an additional 500 bp product [35, 36].

## 5. Conclusion and Future Perspective

The present study supports the historical assumption that *M. bovis* could establish itself in a rhinoceros population and other wildlife but remain underestimated and unrecognized for decades. TB in rhinoceros within a given reserve or facility is a potential risk for human infection, either visitors or workers. Thus, the application of effective tools to determine the tuberculosis status in the rhinoceros is crucial. An organized approach to disease management shared between wildlife and cattle needs to be identified as a key requirement in national and international zoological parks. Integrating these components allows for adaptive disease management and may be the most effective way to manage *M. bovis*. A large-scale study is required to determine *M. bovis* prevalence in the zoological parks of Pakistan and rest of countries.

## Figures and Tables

**Figure 1:** Photographs of one-horned female rhinoceros died of *M. bovis* infection. (a) Showing blood mixed exudate coming out of the vagina (white arrow), (b) uterine pus mixed with tissue debris (blue arrow), (c) small multifocal tubercular lesions (arrowheads) containing creamy white exudate in the lungs, and (d) small multifocal tubercular lesions (arrowheads) on the parietal surface of liver (arrowheads).

**Figure 2:** Photomicrographs of lungs of one-horned female rhinoceros died of *M. bovis* infection showing (a) thickened alveolar septa (double-sided arrows), and alveoli filled with fibrino-necrotic edema (fne) fluid along with massive infiltration of inflammatory cells, (b) micronodules with minimum calcified exudate surrounded by fronts of fibroblasts, fibrocytes, monocytes, macrophages (arrows), multinucleated giant cells, and calcified centre (cc) along with inflammatory cells infiltration in bronchioles (if), (c) two calcified (ca) tubercle nodules surrounded by fronts of fibroblasts, fibrocytes, monocytes, macrophages (arrows), and (d) calcified (ca) centre. H & E; magnification: (a)–(c) 100X; (d) -400X.

**Figure 3:** Photomicrograph of lung tissues of rhinoceros died of *M. bovis* infection showing (a) extensive fibrosis, presence of bacilli (arrows), and hyperplasia of pneumocytes. H & E; 400X. (b) Confirmation of *Mycobacterium bovis* by PCR (500 bp) from lungs (5), liver (6), and uterine pus (7). Lane 1 shows DNA marker (50 bp), lane 3 positive samples and lane 2 and 4 show negative control.

## Data Availability

All the data relevant to this study is mentioned in the manuscript. There is no any supplementary data.
